# Umbilical Cord Mesenchymal Stem Cells Ameliorate Premature Ovarian Insufficiency in Rats

**DOI:** 10.1155/2022/9228456

**Published:** 2022-05-30

**Authors:** Meiliang Zhang, Tingting Xie, Weiyou Dai, Bo Zhao, Yaqin Zheng, Jianmiao Hu, Ruolang Pan, Liang Wang

**Affiliations:** ^1^Department of Obstetrics and Gynecology, The Second Affiliated Hospital, Zhejiang University School of Medicine, Hangzhou, Zhejiang, China; ^2^Department of Obstetrics and Gynecology, Yiwu Maternity and Children Hospital, Yiwu Branch of Children's Hospital, Zhejiang University School of Medicine, Yiwu, Zhejiang, China; ^3^Department of Obstetrics and Gynecology, The Women and Children Hospital of Dongyang, Dongyang Branch of Xinhua Hospital, Shanghai Jiao Tong University School of Medicine, Dongyang, Zhejiang, China; ^4^Provincial Key Laboratory of Cell-Based Drug and Applied Technology Development, S-Evans Biosciences, Institute for Cell-Based Drug Development of Zhejiang Province, Hangzhou, Zhejiang, China

## Abstract

Premature ovarian insufficiency (POI) or premature ovarian failure (POF) is known as a state of hypergonadotropic hypogonadism. Stem cell therapy is expected to be used in the treatment of POI. The aim of the present study was to explore the feasibility and effectiveness of umbilical cord mesenchymal stem cell (UCMSC) transplantation for the treatment of POI in a rat model of POI induced by cyclophosphamide (CTX) injection. The ovarian function was examined by evaluating the weight of the ovary and body, estrus cycle, ovarian morphology, hormonal secretion, granulosa cell apoptosis, and fertility. The results showed that the ovarian function indicators of the modeled rats were comparable to those of the control rats after UCMSC transplantation, indicating that the ovarian function of the modeled rats recovered to a satisfactory extent. Our research may provide an experimental clue for the clinical application of UCMSC transplantation in the treatment of POI. Further experiments will focus on the detailed signaling pathway study of the molecular mechanisms of injury and repairment on the treatment with UCMSCs transplantation in the rat POI models.

## 1. Introduction

Premature ovarian insufficiency (POI), or premature ovarian failure (POF), is known as a state of hypergonadotropic hypogonadism characterized by amenorrhea, hypergonadotropism, and hypoestrogenism [1, 2]. The diagnosis of POI can be made in women younger than 40 years with high follicle-stimulating hormone (FSH) and low estradiol levels assessed in two separate settings at least one month, with amenorrhea lasting for 4 to 6 months [3]. Although many influencing factors of POI have been reported, including genetic, autoimmunologic and infectious factors or chemoradiation histories, the exact cause of POI remains largely unknown in many cases [4–6].

Hormone replacement therapy can alleviate the clinical symptoms of estrogen deficiency. However, it can neither inhibit the FSH rise nor effectively restore the ovarian function; rather, it has some obvious adverse effects [7, 8]. Currently, ovarian tissue transplantation is the only reliable method for the treatment of POI by restoring the endocrine function and fertility of patients [9, 10]. Autologous transplantation is mainly used for patients with the cryopreserved ovarian tissue before chemotherapy or radiotherapy [11–13]. For allogeneic transplantation, rejection is inevitable, and many couples cannot accept ova donation due to cultural and religious reasons [14]. Even successful ovarian transplants do not guarantee fertility [11, 15]. Failure of repeated treatments is the source of physical and mental suffering for patients.

Stem cell therapy seems to be expected to bring substantial benefits to patients suffering from a wide range of diseases and injuries [16]. During embryonic development, mesoderm cells can differentiate into different tissues. After birth, these pluripotent stem cells exist in the organism in the form of mesenchymal stem cells (MSCs) and can maintain their developmental potentiality even after subculture *in vitro* [17]. It has been demonstrated that injecting MSCs cultured *in vitro* into the body and locality for differentiation can achieve tissue regeneration in animal models [14]. The use of MSCs from different sources for POI treatment has achieved positive outcomes in animal models [7, 18, 19]. The transplanted MSCs can differentiate into oocytes and granulosa cells, or restore the ovarian function through paracrine pathways [14, 20]. Clinical trials using MSCs to treat POI have been carried out, but the specific treatment plan and effectiveness need to be further verified [21–24].

The umbilical cord is a source of MSCs for cell therapy [1]. The aim of the present study was to evaluate and compare the therapeutic efficacy of different options of umbilical cord mesenchymal stem cell (UCMSC) transplantation for the treatment of POI in rat models, hoping that the obtained results could provide new potential treatment strategies for POI.

## 2. Materials and Methods

### 2.1. Animal Models

Forty-eight adult Sprague Dawley (SD) female rats weighing 200 ± 10 g were provided by the Animal Center Laboratory of Zhejiang University (Hangzhou, China). All experimental protocols were approved by the Institutional Animal Care and Use Committee of Zhejiang Center of Laboratory Animals (Hangzhou, China) (ZJCLA-IACUC-20050016). These animals were kept under light control (light/dark cycles 12 h each) at 22 ± 2°C room temperature and 55%–60% humidity. After a-week acclimatization, the 48 rats were divided into two groups: (1) a model group (*n* = 36), where the animals received an intraperitoneal (i.p.) injection of 50 mg/kg cyclophosphamide (CTX) (Sigma-Aldrich, St. Louis, MO, USA) on the first day and subsequently 8 mg/kg/day for 14 consecutive days; and (2) a control group (*n* = 12), where the animals received an *i.p.* injection of 0.9% normal saline (NS) instead of CTX [25].

### 2.2. Stem Cell Transplantation

After two weeks of modeling, cell transplantation treatment began. The human UCMSCs preparation and related materials and samples were obtained from S-Evans Biosciences, Ltd. (Hangzhou, China), with the following cluster designation antigens (phenotype) (according to the supplier): CD73^+^, CD90^+^, CD105^+^, CD11b^−^, CD14^−^, CD19^−^, CD34^−^, CD45^−^, and HLA-DR^−^. The 36 animals in the model group were further equally randomized into three groups: a POI group, a UCMSC-iv (intravenous) group, and a UCMSC-OI (ovary injection) group. Prior to UCMSC transplantation, the rats were anesthetized with 3% pentobarbital sodium (50 mg/kg bw). In UCMSC-iv group, UCMSCs were suspended in 100 *μ*L phosphate-buffered saline (PBS) at a concentration of 1 × 10^6^/mL and injected into the tail vein. In UCMSC-OI group, rats were subjected to laparotomy. The injection concentration of UCMSCs was 2 × 10^6^/mL, and each ovary was injected 25 *μ*L [18]. The surgical procedures were done under strict aseptic conditions, and postoperative recovery of the animals was under a red lamp to keep the animals warm. The animals in both control and POI groups received 100 *μ*L PBS injection via the tail vein. In the pilot experiment, there was no significant difference in ovarian injection and tail vein injection of PBS between the control and POI groups.

After the above operation, the 12 rats in each group were equally randomized into two subgroups: one for the treatment experiment and the other for the breeding experiment.

### 2.3. Weight Observation

The rats were weighed at days 0, 7, 14, and 28 after CTX injection, and changes in body weight before and after drug administration were observed.

### 2.4. Examination of the Rat Estrus Cycle

The normal rat estrus cycle usually includes four consecutive stages: P (pre-estrus), E (estrus), M (metestrus), and D (diestrus) [26]. Vaginal smears of rats were taken daily at about 8.00 AM, and the estrus cycle was observed. Specific steps were as follows: a, pressing the back of the rat and lifting the tail up; b, inserting a cotton swab moistened with 0.9% NaCl into the rat's vagina to a depth of about 1–2 cm, turning the swab gently before withdrawal, and evenly spreading the vaginal exfoliated cells on a clean glass slide; and c, drying the smear in air naturally and then pap-staining it to observe the presence of leukocytes, keratinized epithelial cells, and nucleated epithelial cells under a microscope.

### 2.5. Treatment Experiment

Two weeks after stem cell transplantation, the rats used for the treatment experiment were sacrificed by *i.p.* injection of 3% pentobarbital sodium [27]. The blood sample was collected from the inferior vena cava, and both ovaries were removed.

#### 2.5.1. Hormone Assay by ELISA

The blood samples were centrifuged to extract the serum and stored a 20°C for the measurement of biochemical indices, including estradiol (E2), follicle-stimulating hormone (FSH), anti-Müllerian hormone (AMH), and luteinizing hormone (LH) using ELISA kits (Shanghai Enzyme-linked Biotechnology Co., Ltd., Shanghai, China). The sensitivity of the assay was 0.18 ng/mL, 60 pg/mL, 1 ng/mL, and 0.94 mIU/mL for AMH, E2, FSH, and LH, respectively. The intra-assay and inter-assay variation coefficients for AMH, E2, FSH, and LH were all less than 10%.

#### 2.5.2. Ovarian Weight, Follicle Count, and Histopathology Evaluation of Ovarian Tissues

After stripping off the excess fat tissue, the ovaries were weighed to assess the change of ovarian weight index. The ovarian weight index was calculated by comparing the ovarian weight (g) with the body weight (g). Subsequently, the ovaries were immediately fixed with 4% paraformaldehyde in PBS (pH = 7.4), embedded in paraffin, and serially sliced into 5 *μ*m sections. Every fifth section of every ovarian tissue was mounted on glass slides, stained with hematoxylin-eosin (HE). From these sections, the numbers of healthy primordial, primary, secondary, and antral follicles were counted as described previously [28–30]. In every fifth ovarian section, primary, secondary, and antral follicles were counted when the oocyte with nucleus and nucleolus was present in the follicular cross section. Primordial follicles were also counted every fifth section when the oocyte with multiple nucleoli was visible in the follicular cross section [31]. The distribution of ovarian follicular development was evaluated under an optical microscope (DM3000LED, Leica, Germany).

#### 2.5.3. Stem Cell Location by Immunohistochemistry (IHC)

UCMSCs transferred in the ovarian tissue were detected by IHC as described previously [32]. Briefly, the paraffin-embedded sections of the ovarian tissue were deparaffinized and blocked with 5% goat serum for 1 h at room temperature, and then incubated with anti-human mitochondria antibody (Boster Biological Technology Co., Ltd., Wuhan, China) at 4°C overnight. After washing thrice with PBS, the sections were incubated with HRP-conjugated anti-mouse IgG (Beyotime Institute of Biotechnology, Shanghai, China) according to the manufacturer's instructions. The sample was finally stained with DAB reaction, HE counterstained, and photomicrographed under a microscope. Positive expressing cells were counted every fifth section of every ovarian tissue. As controls for immunostaining procedures, some sections were incubated with normal mouse IgG or PBS in place of the primary antibodies. No false-positive reaction was detected in the sections.

#### 2.5.4. Apoptosis Assay by TUNEL

Fragmented DNA was detected histochemically as the indicator of cell apoptosis in the rat ovaries using the TUNEL detection kit (Boster Biological Technology Co., Ltd., Wuhan, China). The paraffin-embedded sections of the ovarian tissue were deparaffinized, rehydrated with ethanol (100%, 90%, 80%, and 75%) in sequence, washed thrice with PBS for 5 min, and incubated with proteinase K at 37°C for 30 min. Subsequently, the diluted biotinylated digoxigenin antibody was added. Fluorescence was used for development. The nucleus was stained with corresponding 4′,6-diamidino-2-phenylindole/hematoxylin. Follicles were considered apoptotic when showing ≥20% TUNEL-positive granulosa cells [33]. The proportion of total atretic follicles was observed in the ovary.

### 2.6. Breeding Experiment

Adult male rats of the same strain were selected for the breeding experiment. Two weeks after stem cell transplantation, the animals were caged at a ratio of 1 male to 2 females for 1 week following the Harem theory. The rats were caged at 5 : 00 pm at the first day, and vaginal smears were performed at 9 : 00 AM on the following day to confirm the mating results. After successful mating, the animals were no longer co-caged. Two weeks later, the female rats were sacrificed and the uterus was collected. The fetuses in rats were counted, and their development was observed.

### 2.7. Statistical Analysis

Data were expressed as the mean ± standard deviation and analyzed using SPSS 20.0 for Windows. Differences between multiple groups were analyzed by one-way analysis of variance (ANOVA) and least-significant difference (LSD) *t*-test. A *p* value less than 0.05 was considered statistically significant.

## 3. Results

### 3.1. Effect of UCMSC Transplantation on Body Weight

Changes in body weight after CTX administration are shown in Figure 1. The weight in the control group in different days was increased steadily (*p* > 0.05), and significances were found in POI, UCMSC-iv, and UCMSC-OI groups after UCMSC transplantation (*p* > 0.05*vs.* control group). Further, the weight in POI group decreased significantly. Compared with POI group, the body weight in UCMSC-iv and UCMSC-OI groups was significantly increased after UCMSC transfer (*p* > 0.05).

### 3.2. Change of the Rat Estrus Cycle

The abnormal degree of the estrus cycle was classified as follows: type I—normal; type II—regular cycle with a shortened estrus; type III—irregular cycle, persistent estrus, or prolonged estrus; and type IV—no periodicity (Figure.  2(a)). Most of the normal rats showed type I, while the rats after CTX injection all showed type IV (Figure.  2(b)). After UCMSC transplantation, types II and III were observed in UCMSC-iv and UCMSC-OI groups (Figure 2(c)). The vaginal exfoliated cells of various rat estrous cycles were displayed in Figure 2(d) by pap-staining. The aforementioned findings indicate that UCMSC transplantation affected the already disordered estrus cycle in rats.

### 3.3. Change in Serum Hormone Level after UCMSC Transplantation

The results of hormone analysis are shown in Figure.  3. Significant differences among the control, POI, UCMSC-iv, and UCMSC-OI groups were found for FSH, LH, AMH, and E2 (all *p* < 0.05). The serum levels of AMH and E2 were significantly decreased, and the serum levels of FSH and LH were significantly increased in POI group relative to controls (*p* < 0.05). These results indicate that the POF animal model was established successfully. Compared with POI group, the serum hormone levels in UCMSC-iv and the UCMSC-OI groups were significantly different and were closer to the control group (*p* < 0.05), demonstrating that UCMSC transfer improved the hormonal disorder of POI.

### 3.4. Changes in Ovarian Weight Index

Significant difference among the control, POI, UCMSC-iv, and UCMSC-OI groups was found (*p* < 0.05). Compared with the control group, the ovarian weight index in POI group was significantly reduced. Compared with POI group, the ovarian weight index in UCMSC-iv and UCMSC-OI groups was significantly increased (*p* < 0.05) (Figure.  4).

### 3.5. Histopathological Findings

Differences for the number of follicles at different stages of development in the control, POI, UCMSC-iv, and UCMSC-OI groups were analyzed, and there was statistical significance (all *p* < 0.05). In the control group, the healthy ovary was observed containing a large number of primordial and primary follicles (Figure 5(a)). In contrast, the number of primordial, primary, secondary, and antral follicles was decreased in the ovaries of POI group (Figure 5(b)). Compared with POI group, the number of healthy primary and secondary follicles in the ovarian slices of UCMSC-iv and UCMSC-OI groups was significantly increased, the shape was more regular, and more antral follicles before ovulation were observed (Figures 5(c) and 5(d)).

According to the number of follicles at different stages (Figures 5(e)–5(h), in POI group, the number of primordial, primary, secondary, and antral follicles was significantly different from that in the control group (*p* < 0.05). Compared with POI group, the number of primordial, primary, and antral follicles was increased in UCMSC-iv group or UCMSC-OI group (*p* < 0.05). For the number of secondary follicles, only UCMSC-OI group had a significant difference compared with POI group (*p* < 0.05).

### 3.6. UCMSCs Infiltrated into the Ovarian Tissue

IHC showed the spatial location of the transferred human UCMSCs in the ovary tissue. Cells with positive staining were observed in the stroma of the ovary tissue in UCMSC-iv and UCMSC-OI groups. However, no UCMSCs were detected in the control and POF groups (Figure 6). The results showed that the number of UCMSC in the UCMSC-iv group was not significantly different from that in the UCMSC-OI group (179.7 ± 27.3 *vs.* 194.3 ± 20.1, *p* < 0.05).

### 3.7. Effect of UCMSC Transplantation on Ovarian Cell Apoptosis

Differences for the percentage of atretic follicles among the control, POI, UCMSC-iv, and UCMSC-OI groups were analyzed by one-way ANOVA (*p* < 0.05). After CTX injection, significantly larger numbers of apoptotic cells (FITC-positive or brown cells) were observed in the ovarian tissue of POI group as compared with the control group (*p* < 0.05) (Figure 7(a)). According to the statistical results, the percentages of atretic follicles in the ovarian sections of UCMSC-iv and UCMSC-OI groups were reduced compared with that in POI group two weeks after UCMSC transplantation (*p* < 0.05) (Figure 7(b)).

### 3.8. Effect of UCMSC Transplantation on Fertility

The mating success rates of animals in the control, POI, UCMSC-iv, and UCMSC-OI groups were monitored and recorded. The recorded results showed that the mating success rate of animals in POI model group was 50% *vs.* 83% in UCMSC-iv group and 100% in UCMSC-OI group (Figure 8(a)). The number of fetuses among the control, POI, UCMSC-iv, and UCMSC-OI groups was analyzed (*p* < 0.05). The statistical results of the number of fetuses showed that the mean number of fetuses per rat in the POI model group was significantly decreased in comparison with that in the control group (*p* < 0.01), whereas the number of fetuses in UCMSC-iv and UCMSC-OI groups was increased (*p* < 0.05*vs.* POI group). In addition, compared with the UCMSC-iv group, the number of fetuses in UCMSC-OI group was significantly increased (*p* < 0.05) (Figure 8(b)). There were no statistical differences between the UCMSC-OI and control groups (*p* > 0.05). No obvious developmental abnormalities were observed in any fetus, suggesting that UCMSC transplantation can significantly improve the fertility of POI model animals.

## 4. Discussion

Although the advancement in anticancer treatment including cytotoxic chemotherapy, radiotherapy, and bone marrow transplantation therapy has greatly improved the survival of cancer patients, they have also brought about POI in women cancer patients [34, 35]. The ovarian function mainly falls into two categories: one is the endocrine function, which can secrete hormones that can affect the growth and development of organs (such as the ovary) and the entire body, and the other is fertility, including the ability to mate successfully and breed healthy pups [4, 18, 36]. According to the previously reported protocol [20, 37], we used CTX to establish a chemotherapy-induced POI rat model to explore the therapeutic effect of UCMSC transfer. The experimental results showed clear ovarian damage in POI group, including changes in ovarian and body weight, estrus cycle, hormone levels, number of follicles, mating, and fertility. After UCMSC transplantation, some parameters were improved, suggesting that UCMSC treatment could alleviate ovarian injury and improve the ovarian function in rats with chemotherapy-induced POI.

Some studies [27, 38] reported that human MSCs had the low expression of human leukocyte antigen major histocompatibility complex I (MHC I) and the absence of MHC II molecules, and could secrete immune-suppressive cytokines in their adjacent microenvironment such as interleukin 10 (IL-10) and transforming growth factor (TGF)-*β*1 without eliciting host immune rejection. They believed that UCMSCs also had these advantages [32]. As UCMSCs can be isolated from the human umbilical cord in large quantities, expanded in culture, frozen/thawed, and engineered, they are considered to be an unlimited source of stem cells [4, 39–41]. Although human UCMSCs have the ability to differentiate into germ cells, recent theories and reports tend to believe that they have yet actually changed in the body [42]. Previous studies [43, 44] have shown that human UCMSCs will not differentiate into follicular structures after transplantation into animals. It may enhance the environmental factors around the ovaries to promote the functional recovery of the injured ovaries [45]. In this study, we found that 14 days after transplantation, human UCMSCs mainly appeared in the rat ovarian interstitium with a limited number, and found that these rats eventually produced normal fetuses, which to a certain extent demonstrated that these implanted cells would not differentiate and cause genetic mixing. In terms of signaling pathways, some current studies [46–49] have shown that UCMSCs could affect ovarian development, follicular growth, and granulosa cell proliferation and differentiation through the Hippo, TGF-*β*1/Smad3, PI3K/Akt, and AMPK/mTOR signaling pathways. Zhao et al. [50] studied the metabolomics of human UCMSCs in the treatment of POI in mice and found that human UCMSCs activated the PI3K pathway by promoting free amino acid levels to restore ovarian function, consequently improving lipid metabolism and reducing the monosaccharide concentration. The action mechanism of UCMSCs in the body is very complex, and related research can better support its clinical application, which is worthy of further study.

The ovarian health is closely related to hormone secretion in the hypothalamic-pituitary-ovarian axis [51, 52]. FSH and LH are gonadotropins, secreted by the pituitary gland responsible for promoting the growth and maturation of follicles [53]. E2 is produced by theca cells and granulosa cells in follicles, and its rising expression level provides negative feedback on pituitary FSH secretion in the hypothalamus-pituitary-ovary axis [19]. AMH is secreted by the granulosa cells of primary and secondary follicles, and inhibits the initiation of the growth of primordial follicles, which is an effective marker of ovarian reserve [54, 55]. Ovarian tissue fibrosis and follicular development disorders are the basic pathological changes of POI [47]. It was found in our study that the number of follicles was reduced, the number of atretic follicles was increased, and granulosa cells were apoptotic in POI group, which led to a decrease in serum levels of AMH and E2. And then, the body regulated the increase of gonadotropins to stimulate follicle growth. However, due to the reduced number of follicles, this stimulation will further deplete the follicles. After UCMSC transplantation, the number of follicles was increased, the number of apoptotic granulosa cells was decreased, and the serum level of AMH and E2 was increased, suggesting UCMSCs could improve the environment around the follicles and inhibit the apoptosis of granulosa cells, thereby promoting the recovery of the ovarian function. All these findings are consistent with previous studies [47, 50].

To explore an optimal stem cell transplantation protocol, we also compared tail vein injection and ovarian injection. It was found that tail vein injection caused less damage and more flexibility in formulating overall treatment plans. It has been reported that i.v. injection of human UCMSCs could promote repair of multiple organs damaged by chemotherapy [1]. Interestingly, comparison of the two injection approaches showed no statistical significance except for the mean number of fetuses. We hypothesize that there are two main possible factors contributing to these results. One factor is time. Two weeks after UCMSC transplantation, the rats used for the treatment experiment are sacrificed, but those for the breeding experiment were still alive. The second factor is the concentration. The cell transplant concentration used in this study may not be optimal. Therefore, in subsequent experiments, we will extend the observation time after cell transplantation and test the therapeutic effects of different cell concentrations on POI rats.

## 5. Conclusion

Our work has demonstrated that UCMSCs can significantly improve the abnormal state of hormone levels in POI rats, promote the growth and development of follicles, and inhibit excessive follicular atresia and granulosa cell apoptosis. UCMSCs should be considered as a valuable source of stem cells that can be used to restore fertility potential. Further experiments will focus on the detailed signaling pathway study of the molecular mechanisms of injury and repairment on the treatment with UCMSCs transplantation in the rat POI models.

### 5.1. Limitation

Our investigation has some limitation. To some extent, the innovation of our experiment was not advanced, because we pay more attention for the confirmatory experimental results. The action mechanism of UCMSCs in the body is very complex, related research can better support its clinical application, and our next study will focus on this.

## Figures and Tables

**Figure 1:** Comparisons of rat body weight in each group. Comparisons among all the groups were examined by one-way ANOVA first, LSD *t*-test was further applied to detect the difference between two groups, and significance was shown. (a) *p* < 0.05*, UCMSC-iv vs. POI;* (b) *p* < 0.05, UCMSC-OI *vs.* POI.

**Figure 2:** Effects of modeling and UCMSC transplantation on rat estrus cycle. (a) Four patterns of abnormal estrus cycles; (b) proportion of various rat estrous cycle patterns in the control and model groups; (c) proportion of various rat estrous cycle patterns in each group after UCMSC transplantation; and (d) *the vaginal exfoliated cells of various rat estrous cycles* (pap-staining, ×200). *Black scale bar = 100 μm.* P*, pre-estrus;* e, estrus; m, metestrus; d, diestrus.

**Figure 3:** The levels of FSH, LH, AMH, and E2 for each group. Differences among the control, POI, UCMSC-iv, and UCMSC-OI groups were detected for FSH, LH, AMH, and E2 using one-way ANOVA, and then comparisons within two groups were examined by LSD *t*-test. (a) FSH; (b) LH; (c) AMH; and (d) E2.  ^*∗*^*p* < 0.05.

**Figure 4:** Comparisons of ovarian weight index in each group. Significance was tested among the control, POI, UCMSC-iv, and UCMSC-OI groups by one-way ANOVA, and comparisons between two groups were further analyzed by LSD t-test. ^*∗*^*p* < 0.05.

**Figure 5:** Ovarian histopathology using HE staining (×20). In different types of follicles, the difference for the number of follicles among the control, POI, UCMSC-iv, and UCMSC-OI groups was analyzed. (a) Control group; (b) POI group; (c) UCMSC-iv group; (d) UCMSC-OI group; (e) counts of primordial follicle; (f) counts of primary follicle; (g) counts of secondary follicle; and (h) counts of antral follicle. Black *scale bar* = 1 mm. ^*∗*^*p* < 0.05.

**Figure 6:** UCMSC location using IHC staining (×400). (a) Control group; (b) POI group; (c) UCMSC-iv group; (d) UCMSC-OI group; (e) isotype control: mouse IgG; and (f) counts of positive cells. Black arrow: human UCMSCs. Black *scale bar* = 50 *μ*m.

**Figure 7:** Cell apoptosis assay. Differences for the percentage of atretic follicles per ovary among the control, POI, UCMSC-iv, and UCMSC-OI groups were analyzed by one-way ANOVA, and comparisons between two groups were further analyzed by LSD *t*-test. (a) Fluorescence results (×200) and (b) percentage of total atretic follicles. White *scale bar* = 100 *μ*m. ^*∗*^*p* < 0.05.

**Figure 8:** Fertility detection. (a) Mating success rate. Differences among the control, POI, UCMSC-iv, and UCMSC-OI groups were analyzed by one-way ANOVA, and further comparisons between two groups were analyzed; and (b) average number of fetuses. Differences among all the groups were analyzed by one-way ANOVA, and comparisons within two groups were further analyzed. ^*∗∗*^*p* < 0.01; ^*∗*^*p* < 0.05.

## Data Availability

The authors will provide raw data to support the conclusions of this research without reservation. The original contributions presented in the study are included in the article, and further inquiries can be directed to the corresponding author.

## References

[1] Zhu S. F., Hu H. B., Xu H. Y. (2015). Human umbilical cord mesenchymal stem cell transplantation restores damaged ovaries. *Journal of Cellular and Molecular Medicine*.

[2] De Vos M., Devroey P., Fauser B. C. (2010). Primary ovarian insufficiency. *Lancet*.

[3] Fazeli Z., Abedindo A., Omrani M. D., Ghaderian S. M. H. (2018). Mesenchymal stem cells (MSCs) therapy for recovery of fertility: a systematic review. *Stem Cell Reviews and Reports*.

[4] Elfayomy A. K., Almasry S. M., El-Tarhouny S. A., Eldomiaty M. A. (2016). Human umbilical cord blood-mesenchymal stem cells transplantation renovates the ovarian surface epithelium in a rat model of premature ovarian failure: possible direct and indirect effects. *Tissue and Cell*.

[5] Jiao X., Ke H., Qin Y., Chen Z. J. (2018). Molecular genetics of premature ovarian insufficiency. *Trends in Endocrinology and Metabolism*.

[6] Liu X. M., Yan M. Q., Ji S. Y. (2018). Loss of oocyte Rps26 in mice arrests oocyte growth and causes premature ovarian failure. *Cell Death & Disease*.

[7] Zhang H., Luo Q., Lu X. (2018). Effects of hPMSCs on granulosa cell apoptosis and AMH expression and their role in the restoration of ovary function in premature ovarian failure mice. *Stem Cell Research & Therapy*.

[8] Rodriguez C., Patel A. V., Calle E. E., Jacob E. J., Thun M. J. (2001). Estrogen replacement therapy and ovarian cancer mortality in a large prospective study of US women. *Journal of the American Medical Association*.

[9] Lee D. M., Yeoman R. R., Battaglia D. E. (2004). Live birth after ovarian tissue transplant. *Nature*.

[10] Silber S. J., Lenahan K. M., Levine D. J. (2005). Ovarian transplantation between monozygotic twins discordant for premature ovarian failure. *New England Journal of Medicine*.

[11] Silber S., Pineda J., Lenahan K., DeRosa M., Melnick J. (2015). Fresh and cryopreserved ovary transplantation and resting follicle recruitment. *Reproductive BioMedicine Online*.

[12] Del-Pozo-Lérida S., Salvador C., Martínez-Soler F., Tortosa A., Perucho M., Giménez-Bonafé P. (2009). Preservation of fertility in patients with cancer (Review). *Oncology Reports*.

[13] Dolmans M. M., Donnez J. (2021). Fertility preservation in women for medical and social reasons: oocytes vs ovarian tissue. *Best Practice & Research Clinical Obstetrics & Gynaecology*.

[14] Wang Z., Wang Y., Yang T., Li J., Yang X. (2017). Study of the reparative effects of menstrual-derived stem cells on premature ovarian failure in mice. *Stem Cell Research & Therapy*.

[15] Donnez J., Jadoul P., Squifflet J., Kim T. (2018). Ovarian tissue cryopreservation and transplantation in cancer patients. *Best Practice & Research Clinical Obstetrics & Gynaecology*.

[16] Trounson A., McDonald C. (2015). Stem cell therapies in clinical trials: progress and challenges. *Cell Stem Cell*.

[17] Chen L., Guo S., Wei C., Li H., Wang H., Xu Y. (2018). Effect of stem cell transplantation of premature ovarian failure in animal models and patients: a meta-analysis and case report. *Experimental and Therapeutic Medicine*.

[18] Song D., Zhong Y., Qian C. (2016). Human umbilical cord mesenchymal stem cells therapy in cyclophosphamide-induced premature ovarian failure rat model. *BioMed Research International*.

[19] Ling L., Feng X., Wei T. (2019). Human amnion-derived mesenchymal stem cell (hAD-MSC) transplantation improves ovarian function in rats with premature ovarian insufficiency (POI) at least partly through a paracrine mechanism. *Stem Cell Research & Therapy*.

[20] Fu X., He Y., Wang X. (2017). Overexpression of miR-21 in stem cells improves ovarian structure and function in rats with chemotherapy-induced ovarian damage by targeting PDCD4 and PTEN to inhibit granulosa cell apoptosis. *Stem Cell Research & Therapy*.

[21] Ding L., Yan G., Wang B. (2018). Transplantation of UC-MSCs on collagen scaffold activates follicles in dormant ovaries of POF patients with long history of infertility. *Science China Life Sciences*.

[22] Igboeli P., El Andaloussi A., Sheikh U. (2020). Intraovarian injection of autologous human mesenchymal stem cells increases estrogen production and reduces menopausal symptoms in women with premature ovarian failure: two case reports and a review of the literature. *Journal of Medical Case Reports*.

[23] Bukovsky A., Caudle M. R. (2021). Immunoregulation of follicular renewal, selection, POF, and menopause in vivo, vs. neo-oogenesis in vitro, POF and ovarian infertility treatment, and a clinical trial. *Reproductive Biology and Endocrinology*.

[24] Yan L., Wu Y., Li L. (2020). Clinical analysis of human umbilical cord mesenchymal stem cell allotransplantation in patients with premature ovarian insufficiency. *Cell Proliferation*.

[25] Shen J., Cao D., Sun J. L. (2020). Ability of human umbilical cord mesenchymal stem cells to repair chemotherapy-induced premature ovarian failure. *World Journal of Stem Cells*.

[26] Wang Z., Wei Q., Wang H. (2020). Mesenchymal stem cell therapy using human umbilical cord in a rat model of autoimmune-induced premature ovarian failure. *Stem Cells International*.

[27] Park HS, Chugh RM, Elsharoud A (2021). Safety of intraovarian injection of human mesenchymal stem cells in a premature ovarian insufficiency mouse model. *Cell Transplantation*.

[28] Meng L., Rijntjes E., Swarts H. (2016). Dietary-induced chronic hypothyroidism negatively affects rat follicular development and ovulation rate and is associated with oxidative stress. *Biology of Reproduction*.

[29] Meng L., Wu Z., Zhao K. (2020). Transcriptome analysis of porcine granulosa cells in healthy and atretic follicles: role of steroidogenesis and oxidative stress. *Antioxidants*.

[30] Myers M., Britt K. L., Wreford N. G., Ebling F. J., Kerr J. B. (2004). Methods for quantifying follicular numbers within the mouse ovary. *Reproduction*.

[31] Meng L., Coleman V., Zhao Y. (2021). Pseudo-starvation driven energy expenditure negatively affects ovarian follicle development. *International Journal of Molecular Sciences*.

[32] Liu Y., Mu R., Wang S. (2010). Therapeutic potential of human umbilical cord mesenchymal stem cells in the treatment of rheumatoid arthritis. *Arthritis Research and Therapy*.

[33] Del Castillo L. M., Buigues A., Rossi V. (2021). The cyto-protective effects of LH on ovarian reserve and female fertility during exposure to gonadotoxic alkylating agents in an adult mouse model. *Human Reproduction*.

[34] Meirow D., Nugent D. (2001). The effects of radiotherapy and chemotherapy on female reproduction. *Human Reproduction Update*.

[35] Green D. M., Sklar C. A., Boice J. D. (2009). Ovarian failure and reproductive outcomes after childhood cancer treatment: results from the childhood cancer survivor study. *Journal of Clinical Oncology*.

[36] Wang S., Yu L., Sun M. (2013). The therapeutic potential of umbilical cord mesenchymal stem cells in mice premature ovarian failure. *BioMed Research International*.

[37] Ling L., Feng X., Wei T. (2017). Effects of low-intensity pulsed ultrasound (LIPUS)-pretreated human amnion-derived mesenchymal stem cell (hAD-MSC) transplantation on primary ovarian insufficiency in rats. *Stem Cell Research & Therapy*.

[38] Bieback K., Brinkmann I. (2009). Mesenchymal stromal cells from human perinatal tissues: from biology to cell therapy. *World Journal of Stem Cells*.

[39] Forraz N., McGuckin C. P. (2011). The umbilical cord: a rich and ethical stem cell source to advance regenerative medicine. *Cell Proliferation*.

[40] Fan C., Wang D., Zhang Q., Zhou J. (2013). Migration capacity of human umbilical cord mesenchymal stem cells towards glioma in vivo. *Neural Regeneration Research*.

[41] Liew A., O’Brien T., Egan L. (2017). Mesenchymal stromal cell therapy for crohn’s disease. *Digestive Diseases*.

[42] Ding C., Li H., Wang Y. (2017). Different therapeutic effects of cells derived from human amniotic membrane on premature ovarian aging depend on distinct cellular biological characteristics. *Stem Cell Research & Therapy*.

[43] Asgari H. R., Akbari M., Yazdekhasti H. (2017). Comparison of human amniotic, chorionic, and umbilical cord multipotent mesenchymal stem cells regarding their capacity for differentiation toward female germ cells. *Cellular Reprogramming*.

[44] Park J. H., Hwang I., Hwang S. H., Han H., Ha H. (2012). Human umbilical cord blood-derived mesenchymal stem cells prevent diabetic renal injury through paracrine action. *Diabetes Research and Clinical Practice*.

[45] Mohamed S. A., Shalaby S., Brakta S., Elam L., Elsharoud A., Al-Hendy A. (2019). Umbilical cord blood mesenchymal stem cells as an infertility treatment for chemotherapy induced premature ovarian insufficiency. *Biomedicines*.

[46] Lu X., Bao H., Cui L. (2020). hUMSC transplantation restores ovarian function in POI rats by inhibiting autophagy of theca-interstitial cells via the AMPK/mTOR signaling pathway. *Stem Cell Research & Therapy*.

[47] Cui L., Bao H., Liu Z. (2020). hUMSCs regulate the differentiation of ovarian stromal cells via TGF-*β* (1)/Smad3 signaling pathway to inhibit ovarian fibrosis to repair ovarian function in POI rats. *Stem Cell Research & Therapy*.

[48] Maidarti M., Anderson R. A., Telfer E. E. (2020). Crosstalk between PTEN/PI3K/akt signalling and DNA damage in the oocyte: implications for primordial follicle activation, oocyte quality and ageing. *Cells*.

[49] Li Z., Zhang M., Zheng J. (2021). Human umbilical cord mesenchymal stem cell-derived exosomes improve ovarian function and proliferation of premature ovarian insufficiency by regulating the Hippo signaling pathway. *Frontiers in Endocrinology*.

[50] Zhao Y., Ma J., Yi P. (2020). Human umbilical cord mesenchymal stem cells restore the ovarian metabolome and rescue premature ovarian insufficiency in mice. *Stem Cell Research & Therapy*.

[51] Ruohonen S. T., Poutanen M., Tena-Sempere M. (2020). Role of kisspeptins in the control of the hypothalamic-pituitary-ovarian axis: old dogmas and new challenges. *Fertility and Sterility*.

[52] Shi L., Zhang Y., Dong X. (2022). Toxicity from a single injection of human umbilical cord mesenchymal stem cells into rat ovaries. *Reproductive Toxicology*.

[53] Bosch E., Alviggi C., Lispi M. (2021). Reduced FSH and LH action: implications for medically assisted reproduction. *Human Reproduction*.

[54] Silva M. S. B., Giacobini P. (2021). New insights into anti-Müllerian hormone role in the hypothalamic-pituitary-gonadal axis and neuroendocrine development. *Cellular and Molecular Life Sciences*.

[55] Moolhuijsen L. M. E., Visser J. A. (2020). Anti-müllerian hormone and ovarian reserve: update on assessing ovarian function. *The Journal of Clinical Endocrinology and Metabolism*.

